# Assessment of Condylar Shape through Digital Panoramic Radiograph among Nepalese Population: A Proposal for Classification

**DOI:** 10.1155/2022/6820824

**Published:** 2022-08-09

**Authors:** Abhishek Gupta, Gaurav Acharya, Harender Singh, Sijan Poudyal, Anju Redhu, Peeyush Shivhare

**Affiliations:** ^1^Department of Oral Medicine and Radiology, Chitwan Medical College, Bharatpur, Chitwan 44207, Nepal; ^2^Department of Orthodontics and Dentofacial Orthopedics, KIST Medical College and Teaching Hospital, Lalitpur 44705, Nepal; ^3^Department of Public Health Dentistry, Chitwan Medical College, Bharatpur, 44207 Chitwan, Nepal; ^4^Department of Public Health Dentistry, People's Dental College, 44705, Nepal; ^5^Department of Oral Medicine and Radiology, PGIDS, Rohtak, Haryana 124001, India; ^6^Department of Dentistry, All India Institute of Medical Sciences, Patna 801507, India

## Abstract

**Background:**

Panoramic radiograph is the first and most commonly advised radiograph for screening of temporomandibular joints/condyles. Different shapes of the mandible have been discussed by various authors with no consensus for a definite classification for condyle shape. This study was conducted with the objective to observe various shapes of condyles, symmetry of bilateral condyles, and variations of condyle shapes among males and females.

**Materials and Methods:**

This cross-sectional study was conducted on digital panoramic radiographs available at a tertiary center of Lalitpur from 25.12.2020 to 20.06.2021 after ethical approval from the institutional review board (reference no. 077/078/27). Panoramic radiographs were selected on the basis of inclusion and exclusion criteria, and various shapes of condyles were noted on HP 15 inch flat LED monitor (1280 × 1024). The collected data was analyzed using SPSS (chi-square test: a *p* value of < 0.05 was considered significant). Intra- and interobserver agreement was observed for condylar shapes.

**Results:**

Among the selected 850 panoramic radiographs (1700 condyles), most of them, i.e., 1343 (79%), were round/oval, followed by flattened, i.e., 149 (8.76%), diamond/angled, i.e., 93 (5.47%), crooked finger shaped, i.e., 28 (1.6%), and mixed, i.e., 46 (2.7%), and the least common shape observed was bifid, i.e., 40 (2.3%) (18 (2.1%) left condyle and 22 (2.6%) right condyle).

**Conclusions:**

Six different types of condyle shapes were noted: type I, oval; type II, flat; type III, diamond; type IV, mixed; type V, bifid; and type VI, crooked finger among the study population of Lalitpur.

## 1. Introduction

The TMJ is a ginglymoarthrodial joint, which aids in mastication and speech. Dentists, especially orthodontists and maxillofacial radiologist, need to have a thorough understanding of the anatomy and morphology of the TMJ to distinguish normal from abnormal condition [1, 2]. Panoramic radiograph is the main screening modality for TMJ abnormalities because of low exposure dose and ease of prescription [2–5].

Several authors have discussed about various types of condyle shape in different parts of the world (geographical variations) [2, 6–9]. The most common classification system (which was found/used in most of the previous studies and also with overall highest number of citations) followed in the previous studies was of oval, bird beak, diamond, and crooked finger types of condyles [2, 7, 9–11]. Two of the studies (second highest overall citation) followed different classification as rounded, angled, flattened, and mixed types of condyles [6, 12]. The other two studies followed different classification as round, angled, flat, and convex [13, 14]. One of the study used triangular, round, beak, and flat as classification of condyle [15]. Other used classification as rounded, angled, flattened, and pointed [8]. Most of the previous studies found 4 types of condyles in their study population, and only in one study, 6 types of condyles were found which were round, flattened, diamond, mixed, crooked finger, and bifid. Apart from the most commonly used classification system which was first given by Sonal et al. [2] (Table 1), the other studies found round, angled, and flattened in their study groups.

These variations in shapes of condyles among different study population would not justify using any of the studies for universal classification of condyles. Therefore, we conducted this study on digital panoramic radiograph to identify the types of condyles in our part of the world.

The objective of this study was to (a) evaluate the variation in the shapes of the condyle, (b) compare differences or changes between the shapes of condyles between males and females, and (c) determine the occurrence of symmetry in the shape of the condyle on either side.

## 2. Materials and Methods

This cross-sectional study was conducted in Department of Oral Medicine and Radiology, KIST Medical College and Teaching Hospital, Lalitpur, Nepal, among the subjects who had visited the Department of Oral Radiology for panoramic radiograph requiring various dental treatments from 25.12.2020 to 20.06.2021. Ethical approval was given by the ethical review committee of the same institution with IRC reference no. 077/078/27. Written consent was taken from the patient or patient's guardian before using the radiographs. The criteria for inclusion in this study were panoramic radiographs of patients from the age of 11 years and above with demographic data (age and gender), showing complete mandible view on either side with optimal density and contrast without any image distortion projection errors. Exclusion criteria were panoramic radiographs revealing any pathology (osteomyelitis, osteoporosis, etc.) in the maxilla or mandible or revealing any sign of fracture in the mandible, developmental anomalies of the jaws, syndrome of craniofacial structures, plating for fractures, odontogenic cysts or tumors of the jaws, and complete denture and edentulous dental arches. All available panoramic radiographs from 25.12.2020 to 20.06.2021 were saved in a folder named total panoramic radiograph by the principal investigator, and one by one of the panoramic radiograph images (with panoramic radiograph number only visible) was transferred to another folder named study panoramic radiographs by the investigator 2 (who did not participate in the measurements for the study) on the basis of inclusion and exclusion criteria. Thus, convenience sampling was done, and 850 panoramic radiographs were selected. The sample was grouped according to gender and age categories. Five age groups were identified: 11-20, 21-30, 31-40, 41-49, and >50 years. Panoramic radiographs were recorded for routine investigation by a 9000 digital panoramic and cephalometric system (Carestream, France) at 70 kVp, 10 mA, 14.3 s. The obtained images were analyzed on HP 15-inch flat square LED monitor with 1280 × 1024 screen resolution with fixed contrast and brightness to ensure optimal visualization. The images were calibrated (1 : 1 magnification) before tracing of the condyles. Hundred panoramic radiographs were analyzed by two (for interobserver bias/variability) of the investigators (Nos. 1 and 3) with sufficient light on the monitor, and the observer outlined the condyles using the Tracing version 2020.2.0.0 software. Investigator No. 1 analyzed 100 panoramic radiographs again after 15 days (intraobserver bias/variability). Later, all panoramic radiographs were analyzed by the investigator No. 1.

The collected data was analyzed using SPSS. Chi-square test was performed to check the significance level of associations. The *p* value of < 0.05 was considered significant. Intraobserver agreement of condylar shape, expressed as kappa values, ranged from 0.826 to 0.851 for observer 1 and observer 2. Interobserver agreement for condylar shape, expressed as kappa value, ranged from 0.848 to 0.871. Thus, both intra- and interobserver variability showed very good agreement for all observed condylar shapes.

## 3. Results

Among the selected 850 panoramic radiographs on the basis of inclusion and exclusion criteria, 515 (60.6%) were of males, and 335 (39.4%) were of females. Panoramic radiographs were divided into 5 different groups according to age interval of 10 years. There are 217 panoramic radiographs in group i (11-20 years), 272 panoramic radiographs in group ii (21-30 years), 142 panoramic radiographs in group iii (31-40 years), 91 panoramic radiographs in group iv (41-50 years), and 128 panoramic radiographs in group V (>50 years). A total of 1700 condyles were evaluated (including both left and right condyles on an panoramic radiograph). We found six different shapes of condyles: type I, oval; type II, flat; type III, diamond; type IV, mixed; type V, bifid; and type VI, crooked finger (Figure 1).

Among the 1700 condyles, most of them, i.e., 1343 (79%), were round/oval, followed by flattened, i.e., 149 (8.76%), diamond/angled, i.e., 93 (5.47%), crooked finger shaped, i.e., 28 (1.6%), and mixed, i.e., 46 (2.7%), and the least common shape observed was bifid, i.e., 40 (2.3%) (18 (2.1%) left condyle and 22 (2.6%) right condyle) (Tables 2 and 3).

There was no significant difference between males and females in both the left (*p* value 0.162) and right (*p* value 0.072) condyle shapes (Tables 4 and 5).

739 (82.2%) condyle pairs were symmetric (611 round/oval, 38 flattened, 24 diamond/angles, 7 crooked finger, 8 bifid, and 11 mixed), and 151 were asymmetric.

## 4. Discussion

TMJ is a freely movable articulation between the condyle of the mandible and the squamous portion of the temporal bone at the base of the skull. The TMJ is a ginglymoarthrodial joint, a term that is derived from the ginglymus, meaning hinge joint, allowing motion only backward and forward in one plane, and the orthroid, meaning a joint which permits a gliding motion of the surface [1]. The most important functions of the temporomandibular joint (TMJ) are mastication and speech and are of great interest to dentists, orthodontists, clinicians, and radiologists. This interest stems from the standpoints of structure, function, adaptability, symptomatology, pathology, and imaging [1]. Morphologic changes of the condyle occur due to developmental variations, remodeling, various diseases, trauma, endocrine disturbances, and radiation therapy. Human mandibular condyles may be categorized into five basic types: flattened, convex, angled, rounded, and concave [2].

Other authors have classified the condyle in four types in lateral and posterior view—round, angled, flattened, and mixed type [6]. The only study done in Nepal has identified four types of condylar morphology accordingly: type I, oval shaped; type II, bird beak shaped; type III, diamond shaped; and type IV, crooked finger shaped [7].

We found round/oval shape to be the highest prevalence (79%) in our population which was similarly high in studies done by Khanal (63.6%) [7], Sonal et al. [2] (60%), Anisuzzaman et al. [16] (60%), Maqbool et al. [13] (60.6%), Jawahar and Maragathavalli [11] (58.5%), Shaikh et al. [9] (50%), Kanjani et al. [14] (46.12), Nagaraj et al. [15] (142.8%), Singh and Chakrabarty [12] (41%), Singh et al. [8] (35.4%), and Singh et al. [17] (34.5%). The difference in percentage could be because our study included a very wide range of age group, i.e., as young as 11 years to >50 years of patients, which was not taken with any of the studies.

The second most common shape seen in our study was flattened (8.76%) which was similar to the study by Nagaraj et al. [15] (7.5%), quite higher among the studies by Singh and Chakrabarty [12] (19%) and Singh et al. [17] (14%), quite lower in few of the studies by Singh et al. [8] (2.85%), Maqbool et al. [13] (2.58%), Kanjani et al. [14] (2.62) but reported it to be the most common after diamond/angle shape, whereas studies done by Sonal et al. [2], Khanal [7], Shaikh et al. [9], Anisuzzaman et al. [16], and Jawahar and Maragathavalli [11] did not mention about flattened shapes.

The third most common shape seen in our study was diamond/angled (4.7%), which was similarly seen in other studies by Sonal et al. [ 2] (9%), Singh et al. [8] (3.2%), Shaikh et al. [9] (4.8%), Anisuzzaman et al. [16] (9%), and Jawahar and Maragathavalli [11] (9%), whereas it was quite high in the studies by Khanal [7] (22.64%), Singh and Chakrabarty [12] (28%), Kanjani et al. [14] (29.29), Maqbool et al. [13] (29.31%), and Singh et al. [17] (30.33%). This could be attributed to the reason that these studies have included a bird beak shaped as one of the classification which was not included in our study as well as studies [2, 8, 9, 11] similar to our study. Nagaraj et al. [15] and Singh and Chakrabarty [12] have not discussed about diamond shape in their study.

The fourth most common shape found was the mixed shape of the condyle (3.5%) which was very less than the study done by Singh and Chakrabarty [12] (12%) and Singh et al. [17] (11.16%) whereas other studies [2, 7–9, 13–16] did not mention about mixed shape of condyle.

The least common shape noted in our study was a crooked finger shape (1.2%), almost half more prevalent than the bifid shape (3.16%), which was similarly seen in studies by Singh et al. [17] (1.5%), Anisuzzaman et al. [16] (2%), and Singh and Chakrabarty [12] (2%) higher in other study by Khanal [7] (4.15%), Shaikh et al. [9] (4.8%), and Jawahar and Maragathavalli [11] (14%), whereas most of the other studies did not mention about crooked shaped condyle, and none of the studies mentioned about bifid condyle except one study by Singh et al. [17] (5.33%).

Previous studies have identified mostly 4 different types of condyles, whereas our study found 6 different types, and also, other studies have not included the bifid type in their classification. The differences in our results could be majorly because our study population was entirely different from other studies, and none of the studies had taken a large sample size as ours. As we did our study following the previous studies, we tried to find as many shapes as possible and mentioned in previous studies. Bifid condyle can be detected by panoramic radiograph [18] but to our surprise the bifid condyle which could also have been considered/seen by other researchers as well. Although we agree that the prevalence of bifid condyle is very low (0.31-3.5%) [18–23], its real prevalence has not been predicted yet in our population.

To date, there is no classification for condyle shapes that are accepted uniformly worldwide; therefore, proposing this classification could be considered and accepted. To the best of our knowledge, none of the previous studies have proposed any classification with 6 different types of condyle shapes in their studies; this requires us to propose a classification for condyle shapes. The reason behind this could be that the sample size in previous studies was quite less as compared to our study. This range of variations in condyle shapes could be considered normal and should not be considered an abnormality. This classification will help dentists to identify normal condyle shapes and prevent them from any inadvertent treatment plans. This classification will provide a baseline for future studies as well. This classification can further be used for evaluation of gender and age estimation in forensic dentistry. Limitation of our study was limited samples from one institution, and a convenience sampling method was used.

## 5. Conclusions

Our study concluded that round/oval shape condyle is most commonly seen among the Lalitpur population followed by flat shape, and the least common is crooked finger shape and bifid condyle. We could identify 6 different types of condyle shapes, and we would like to propose a classification of condylar shapes with 6 different types as follows: type I, oval (the upper outer margin/cortical surface of condyle is oval in shape); type II, flat (the upper outer margin of condyle is flattened in shape); type III, diamond (the upper outer margin of condyle is angled/around 90° in shape appearing as tip of diamond); type IV, mixed (the upper outer margin of condyle is not identified as a particular shape); type V, bifid (the upper outer margin of condyle has depression, and a linear cortical line is seen in between the condyle); and type VI, crooked finger (the condyle appears to be slightly bending medially appearing as a crooked finger).

We would suggest for a countrywide study to determine more accurate data on the prevalence of various shapes of condyles among the Nepalese population. Moreover, this study was done using panoramic radiograph (two-dimensional imaging), three-dimensional imaging, or skull study would be more accurate even dimensionally.

## Figures and Tables

**Figure 1:** Six types of condyle shapes.

**Table 1:** Distribution of different classification for condylar shapes and their citations.

Types of condyles	Author (citations)					Total no. of citations
Oval, bird beak, diamond, crooked finger	Sonal V (20)	Khanal P (1)	Shaikh AH (1)	Md Anisuzzaman M (9)	Jawahar A (3)	34
Rounded, angled, flattened, mixed	Ribeiro EC (23)	Singh M (5)				28
Triangular, round, beak, flat	Nagaraj T (6)					6
Round, angled, flat, convex	Maqbool S (5)	Kanjani V (1)				6
Rounded, angled, flattened, pointed	Singh B (3)					3
Round/oval, flattened, diamond/angled, mixed, crooked finger, and bifid	Singh A (0)					0

**Table 2:** Distribution of variations in mandibular right condyle.

Right condyle	Frequency	Percent
Round/oval	674	79.3
Flattened	74	8.7
Diamond/angles	40	4.7
Crooked finger	10	1.2
Bifid	22	2.6
Mixed	30	3.5
Total	850	100.0

**Table 3:** Distribution of variations in mandibular left condyle.

Left condyle	Frequency	Percent
Round/oval	670	78.8
Flattened	75	8.8
Diamond/angles	53	6.2
Crooked finger	18	2.1
Bifid	18	2.1
Mixed	16	1.9
Total	850	100.0

**Table 4:** Distribution of variations in mandibular right condyle among males and females.

Gender	Right condyle shape						Total
	Round/oval	Flattened	Diamond/angles	Crooked finger	Bifid	Mixed	
Male							
No.	263	34	8	4	11	15	335
% within male	78.5%	10.1%	2.4%	1.2%	3.3%	4.5%	100.0%
% within right condyle shape	39.0%	45.9%	20.0%	40.0%	50.0%	50.0%	39.4%
Female							
No.	411	40	32	6	11	15	515
% within female	79.8%	7.8%	6.2%	1.2%	2.1%	2.9%	100.0%
% within right condyle shape	61.0%	54.1%	80.0%	60.0%	50.0%	50.0%	60.6%
Total							
No.	674.0	74.0	40.0	10.0	22.0	30.0	850.0
% within gender	79.3%	8.7%	4.7%	1.2%	2.6%	3.5%	100.0%

**Table 5:** Distribution of variations in mandibular left condyle among males and females.

Gender	Left condyle shape						Total
	Round/oval	Flattened	Diamond/angles	Crooked finger	Bifid	Mixed	
Male							
No.	267	33	12	8	7	8	335
% within male	79.7%	9.9%	3.6%	2.4%	2.1%	2.4%	100.0%
% within left condyle shape	39.9%	44.0%	22.6%	44.4%	38.9%	50.0%	39.4%
Female							
No.	403	42	41	10	11	8	515
% within female	78.3%	8.2%	8.0%	1.9%	2.1%	1.6%	100.0%
% within left condyle shape	60.1%	56.0%	77.4%	55.6%	61.1%	50.0%	60.6%
Total							
No.	670	75	53	18	18	16	850
% within gender	78.8%	8.8%	6.2%	2.1%	2.1%	1.9%	100.0%

## Data Availability

The data supporting the results of this study were obtained from the Department of Oral Medicine and Radiology, KIST Medical College and Teaching Hospital, Lalitpur, Nepal. The data used are included within the article and are also available by email to the corresponding author.
